The article "Promotion of Differentiating Bone Marrow Mesenchymal Stromal Cells (BMSCs) into Cardiomyocytes via HCN2 and HCN4 Cotransfection" was retracted in 2024. Reasons: signs of a paper mill; suspected computer-generated content; unreliable results or conclusions; concerns about the data.

# Promotion of Differentiating Bone Marrow Mesenchymal Stromal Cells (BMSCs) into Cardiomyocytes via HCN2 and HCN4 Cotransfection

**DOI:** 10.1155/2021/5529276

**Published:** 2021-05-13

**Authors:** Xue Luo, Hongxiao Li, Xiaolin Sun, Qisheng Zuo, Bichun Li, Ye Zhu, Wei Wei, Xiang Gu

**Affiliations:** ^1^Medical College of Yangzhou University, Yangzhou, Jiangsu 225001, China; ^2^Department of Pathology, Medical College of Yangzhou Polytechnic College, Yangzhou, Jiangsu 225009, China; ^3^Department of Cardiology, Northern Jiangsu People's Hospital, Yangzhou, Jiangsu 225001, China; ^4^College of Animal Science and Technology, Yangzhou University, Yangzhou, Jiangsu 225001, China

## Abstract

**Aim:**

Investigation of the influences HCN2 and HCN4 has on bone marrow mesenchymal stromal cells (BMSCs) on cardiomyocyte differentiation.

**Methods:**

Miniature adult pigs were used for bone marrow extraction and isolation of BMSCs. The identification of these BMSCs was done by using flow cytometry for the detection of expressed surface antigens CD45, CD11B, CD44, and CD90. Using HCN2 and HCN4 genes cotransfected into BMSCs as group HCN2+HCN4 while myocardial induction solution was used to induced BMSC differentiation in the BMSC induction group. Myocardial marker proteins *α*-actin and cTnT were detected by immunofluorescence staining, while *α*-actin, cTnT, and Desmin myocardial marker proteins expressed were detected by Western blot. The whole-cell patch-clamp technique was used to identify and detect cellular HCN2 channels, HCN4 channel current activation curve, and the inhibitory effect of CsCl on heterologous expression currents.

**Results:**

Flow cytometry results showed that CD45 and CD11B were expressed negatively while CD90 and CD44 were positive. Post HCN2 and HCN4 gene transfection, immunofluorescence staining, and Western blot showed significantly increased HCN2, HCN4, *α*-actin, and cTnT expressed in group HCN2+HCN4 were, which could be compared to the expression levels in the BMSC-induced group. The HCN2+HCN4 group was able to document cell membrane channel ion currents that were similar to If properties.

**Conclusion:**

HCN2 and HCN4 overexpression can considerably enhance the MSC ability to differentiate into cardiomyocytes in vitro and restore the ionic current.

## 1. Introduction

Myocardial infarction (MI) is considered one of the most general and severe types of coronary heart disease present in the elderly [1]. It is mainly caused by narrowing of coronary arteries caused by atherosclerosis, resulting in myocardial ischemia, injury, arrhythmia, heart failure, cardiogenic shock, or sudden cardiac arrest which establishes it as one of the main causes of sudden death in clinical practice [2]. According to results from a survey conducted, the United States has approximately 620,000 new MI patients each year, of which 15% die, unfortunately [3]. At present, MI prevention and treatment revolve mainly around preventive drugs and surgical treatment. Available drugs include aspirin and nitroglycerin; however, most drug solitary helps to relieve pain and is not able to allow for effective improvement of the condition [4]. In terms of surgical treatment, coronary intervention (PCI) or coronary artery bypass grafting (CABG) [5] continues to be the methods that are mainly implemented with evident effects, but long-term drug use is required postsurgery. Therefore, researchers began to construct research along the lines of biological pacemakers with the key strategies including cells and genes. However, this has yet to pass the animal experimental research stage.

Over the past decade, the concept of myocardial regeneration in multiple clinical trials has moved its focus gradually from basic science and animal experiments to bone marrow- (BM-) derived stem or progenitor cells. This includes acute MI and ischemic cardiomyopathy. In the adult bone marrow, in addition to the already well-known hematopoietic stem cells, there are other rare cell populations with powerful differentiation potential and multilineage differentiation function [6]. These cell populations are heterogeneous which include endothelial progenitor cells (EPCs), multipotent mesenchymal stromal cells (MSCs), and multifunctional stem cells (PSCs) that possess a variety of typical markers. More attention has been brought to multifunctional stem cells derived from the bone marrow since they contain cardiomyocyte and vascular endothelial cell differentiating abilities. Among them, MSCs are the most promising source of cellular inflammation and degenerative disease treatment due to their multidirectional differentiation potential and immunoregulatory and proangiogenic characteristics [7]. Early stages of MSCs were discovered to spontaneously differentiate into osteoblasts, chondrocytes, and adipocytes [8]. With the development of research, MSC differentiation potential was discovered to be wider than initially imagined with the ability to produce neuroectoderm- and endodermal-derived cells, including hepatocytes, cardiomyocytes, alveolar neuronal, and intestinal epithelial cells under specific conditions in vitro [9, 10]. Although MSC strong differentiation ability provides to be a new therapeutic agent for regenerative medicine, the safety of transplanted post-MSC unconscious differentiation remains debatable. It has been pointed out that in patients treated with MSC inhibition presented with calcified and ossified encapsulated structures in the infarcted area of the heart [11], visual loss, retinal detachment, and intraocular haemorrhage were also observed in 3 patients that had macular degeneration after adipose tissue-derived MSC (AT-MSC) treatment [12]. Therefore, the directional differentiation of MSCs remains a crucial problem that needs to be solved after cell transplantation.

Studies have shown that the time- and voltage-dependent inward current generated by the hyperpolarized cyclic nucleotide-gated channel (HCN) contributes to the tissue-specific rhythmic activity of the brain and heart [13]. HCN4 and HCN2 are two subtypes of HCN channels, both expressed in the heart [14]. It has been reported that HCN2 and HCN4 synergistically assemble and form functional heterogeneous channels in the Chinese hamster ovary cells (CHO), mouse embryonic heart, and rat thalamus [15]. Er et al. [16] used HCN2 and HCN4 adenovirus vectors to infect neonatal mouse cardiomyocytes, which significantly accelerated the heartbeat. The influence of HCN2 and HCN4 on cardiac pacing was confirmed. In addition, Li et al. [17] found that after rat BMSCs differentiate into cardiomyocytes, they can greatly enhance the pacemaker phenotype, that is, increase the expression of HCN4 and Tbx3/2. However, whether HCN2 and HCN4 can promote the pacing effect of BMSC-differentiated cardiomyocytes has not been reported in the literature. Therefore, in this experiment, we investigated the effects of HCN2 and HCN4 on the differentiation of BMSCs into cardiomyocytes and on cardiac pacing by isolating BMSCs in vitro. It is hoped to provide effective data support for the clinical application of BMSCs in the treatment of MI.

## 2. Materials and Methods

### 2.1. Bone Marrow Stem Cell (BMSC) Extraction

20-40 kg minipigs were used, relatively fixed, and sedated in lateral decubitus position. After this, lidocaine was given at the posterior superior iliac spine for local anaesthesia. Extraction of the bone marrow was performed under bone marrow aspiration with heparin anticoagulation used. The sample obtained was added to the red blood cell lysate, fully vortexed, and mixed. After a 20 min incubation in the dark at room temperature conditions, centrifugation was done at 4°C and 500 r/min for 10 minutes. The supernatant was removed using gentle suction. Red blood cells were lysed in duplicate. Another sterile test tube was obtained with the addition of the Ficoll separating medium before the slow addition of the diluted and mixed bone marrow fluid to the top of the Ficoll separating medium along the wall of the tube. Centrifugation was completed at 2500 r/min for 10 min at 4°C. Postcentrifugation, the second cell layer was slowly sucked and placed into another centrifuge tube and blown and beat evenly with 5 mL PBS before centrifuged again at 1000 r/min for 10 min at 4°C. The supernatant was then gently drawn suck out and added to 2 mL PBS to blow and disperse the cells. The sample was then filtered with a 4 *μ*m filter for cell collection before culturing was done in RPMI 1640 complete medium for future use.

### 2.2. BMSC Surface Antigens Detected by Flow Cytometry

The well-grown BMSC population was selected and consumed with 0.25% trypsin-EDTA digestive juice. The cells were then rinsed with PBS 3 times and centrifuged for 5 min. Resuspension was done with sterile PBS to adjust the concentration to 2 × 10^8^/L. Preparation was then done by adding 1 × 10^6^ cells into individual tubes along with primary antibodies such as mouse anti-mouse porcine CD11B, mouse anti-mouse porcine CD45, mouse anti-mouse porcine CD90, mouse anti-mouse porcine CD44, and mouse IgG negative control (1 : 1000 dilution; all from eBioscience, USA) with a supplementary blank control set at the same time. After incubation at 4°C for 30 min and centrifugation, the upper liquid was removed, and the process was repeated three times to rinse off excess antibody. Washed cells were identified following detection by flow cytometry (Becton Dickinson, USA).

### 2.3. BMSC Differentiation and Grouping

Transmission of BMSCs to the third passage was done with cells collected as the control group. The cells were then plated into 24-well plates plated with Matrigel and cultured until the confluence was 80%~90%. Lentivirus-coated HCN2 and HCN4 overexpression vectors constructed by GenePharma (Shanghai, China) were transfected into BMSCs simultaneously under strict accordance with instructions. The fresh conventional medium was replenished after 12 hours. After 48 hours of continued culturing, the cells were collected and marked as group HCN2+HCN4. Cardiomyocyte induction solution (10 *μ*mol/L 5-Aza+serum-free 1640 medium) was then added wells with cardiomyocyte induction solution being replenished every 48 h for 14–21 days. This was then known as the BMSC induction group. Postinduction completion, cell morphology of the individual group was observed.

### 2.4. Immunofluorescence Staining

The isolated BMSCs also known as treated cells were rinsed 3 times with PBS for 10 min each. 4% paraformaldehyde was then added to the cells for a 30-minute fixation before paraformaldehyde was absorbed and discarded and rinsed 3 times with PBS. 0.2% TritonX-100 was added to the membrane for permeabilization for 20 min. This was then followed by rinsing 3 times with PBS and treatment with 10% FBS for blocking for 2 hours. Blocking solution was extracted and discarded before the addition of primary antibodies HCN2, HCN4, *α*-actin (Abcam, UK), and cTnT (Abcam, UK) proteins in different wells, respectively, overnight. Subsequently, the corresponding secondary antibody was added and incubated for 2 hours in the dark, rinsed in PBS for 3 times, and stained with DAPI for 2 min.

### 2.5. Western Blot

24-well plates were used to implant treated at 2.5 × 10^4^ cells per well in three replicate wells per group. After 24 hours of conventional medium culturing, trypsin digestion was used to collect cells. RIPA protein lysate was implemented to extract total protein with protein concentration determined by BCA. SDS-PAGE electrophoresis was then applied for protein separation before being transferred to PVDF membranes. Blocking for 2 h at room temperature was then employed following with primary antibodies *α*-actin (Abcam, UK), cTnT (Abcam, UK), and Desmin (Abcam, UK) incubation at 4°C overnight. Secondary antibodies were added the next day and incubated for 1 h at room temperature. After rinsing 3 times and dropping the developer on the membrane, it was placed in a gel imaging system for exposure and photography. The gray values of the target protein bands were examined by ImageJ software using *β*-actin as an internal reference.

### 2.6. Whole-Cell Patch-Clamp Technique

The whole-cell patch-clamp technique was used to detect the activation curve of HCN2 and HCN4 channel currents along with the inhibitory effect of CsCl on heterologous expression currents in group HCN2+HCN4 cells. The cells with positive transfection were digested with 0.25% trypsin and implanted on the cell plate. Following complete attachment, a single stem cell with stable attachment, complete cell contour, and green fluorescence was selected under the fluorescence microscope for practical testing. A micromanipulator was used to slowly approach the glass microelectrode to the cell. The glass microelectrode was gently pressed in the centre of the cell and gently given a glass microelectrode for negative pressure suction. The electrode tip then waited for the cell membrane to indicate a high resistance sealing above 1 G*Ω* formation to compensate for the electrode capacitance. After around 1 min, the pulsed negative pressure was gently applied to the glass microelectrode to break the membrane, so that the cell could directly communicate with the internal solution of the electrode and insulate from the extracellular fluid. The whole-cell recording model was constructed with the ion current which was recorded.

### 2.7. Statistical Analysis

SPSS 24.0 software was applied for one-way analysis of variance and independent sample *t*-test analysis with the statistical data as expressed as mean ± standard deviation (SD). An indication of a statistically significant difference was *P* < 0.05.

## 3. Results

### 3.1. Porcine Bone Marrow BMSC Isolation and Identification

Bone marrow aspiration was used to collect porcine bone marrow for BMSC isolation. The flow cytometry results (Figure 1) showed that BMSCs expressed CD45 and CD11B negatively, while CD90 and CD44 were positive (90%). From the results gained, it can be confirmed that the cultured porcine bone marrow stem cells followed stem cell characteristics.

### 3.2. In Vitro Differentiation of BMSCs to Cardiomyocytes Could Be Considerably Increased by HCN2 and HCN4

To determine the effect of expressed HCN2 and HCN4 on BMSC cardiomyocyte differentiation, we first overexpressed HCN2 and HCN4 in BMSCs. When observing the immunofluorescence staining results, BMSC-induced fluorescence expression of HCN2 and HCN4 was higher than that of BMSC induced, indicating successful establishment of the HCN2+HCN4 cotransfected cell group (Figure 2).

Immunofluorescence staining was used to detect further cardiomyocyte marker protein *α*-actin and cTnT expression. The results showed that BMSC induced a noteworthy rise in of *α*-actin and cTnT in HCN2+HCN4 fluorescence expression compared with the BMSC group with consistent *α*-actin and cTnT expression in the HCN2+HCN4 BMSC myocardial induction group (Figure 3(a)). Meanwhile, the results of Western blot showed that the expression of HCN2+HCN4 *α*-actin, cTnT, and Desmin was knowingly amplified in the BMSC-induced group compared with the BMSC group with the consistent protein expressed in the HCN2+HCN4 BMSC-induced group (Figure 3(b)). This shows that the increased expression of HCN2 and HCN4 can directionally induce differentiation of BMSCs into cardiomyocytes.

### 3.3. HCN2 and HCN4 Restored Ionic Currents in BMSC Cultured In Vitro

The results of patch-clamp experiments display that the HCN2+HCN4 group was able to record ion currents in cell membrane channels that are If characteristic alike. This current has the characteristics of hyperpolarization-clamped voltage activation and time dependence with fit responses to intracellular cAMP that are consistent with the typical characteristics of the If pacing current (Figure 4(a)) and currently blocked by CsCl treatment (Figure 4(b)).

## 4. Discussion

MSCs possess the potential for indeterminate differentiation. Numerous experiments regarding the transplantation of MSCs for disease treatment have been carried out revealing various problems throughout the experimental progress. Autologous transplantation of MSCs in patients with the fulminant disease is difficult due to extensive cell preparation periods and transplantation time. MSCs are termed allogeneic transplantation studies due to their lack of costimulatory molecules and major histocompatibility complex (MHC) class II protein expression, which have low immunogenicity [6]. However, complications are still existent in performing allogeneic MSC transplantation, including expressed MHC-class I molecules by allogeneic MSCs, resulting in the activation of allogeneic immune responses and exacerbating persistent inflammation post-MSC transplantation [7]. Additionally, MSC transplantation frequently rises cytomegalovirus (CMV) and herpes simplex virus (HSV) infection risks. Individuals up for MSC transplantation must therefore be screened for CMV and HSV to prevent viral infection in those that are immunosuppressed [9]. However, an insufficient number of studies existing have found MSC-derived secretions have promoting tissue repair and regeneration functions with MSC secretions being rich in a mixture of growth factors for wound healing and neovascularization. These include metalloproteinases- (TIMP-) 1 and 2, and fibroblast growth factor- (FGF-) 6 and 7 [11]. Studies have exhibited that MSC secretions are also able to regulate apoptosis under physiological or pathological conditions. MSC culture supernatant has a reduction in expressed proapoptotic genes Bax and caspase-3 in parenchymal cells while growing in expressed antiapoptotic gene Bcl-2 that played a protective role in parenchymal cells in a constant inflammatory environment [12]. Interestingly, MSC-CM treatment notably declined in breast cancer growth and amplified tumour-bearing mouse survival rates. This altogether indicates that MSC culture supernatant has the ability to extensively inhibit tumour cell viability. Several experimental studies have shown that MSCs have cardioprotective effects on the heart [18]. Then again, MSC-derived secreted proteins, or exosomes (MSC-Exos), can be used for cardiomyocyte regeneration [19]. Huang et al.'s study pointed out that MSC-Exos not only advances cardiomyocyte contractility but also reduces infarct size [20].

Whether it is individually or secretively improving myocardial infarction by MSCs, does not need further discussion. However, the vital problem that needs to be solved is the problem of directional differentiation posttransplantation. Several clinical trials have shown that, based on current immunosuppressive properties of MSCs, finding an appropriate balance between the safety and efficacy of treatment-based therapy is critical in determining the optimal number of transplanted MSCs [20]. However, some patients with idiopathic pulmonary fibrosis (IPF) who received MSC transplantation therapy have developed an infection and respiratory symptoms shortly after, suggesting that MSC-based therapy leads to excessively suppressed immune responses in injured lungs [21]. Similarly, an increase in respiratory and gastrointestinal infections was observed in patients with inflammatory bowel disease (IBD) who had recently taken immunosuppressive drugs ahead of MSC injection [22].

There have been many studies that highlighted that the overexpression of HCN channel-related proteins is a strategy for generating biological pacemakers. Along with the overexpressed HCN2 or HCN4, genes restore ionic currents in mesenchymal stem cells cultured in vitro [23]. Instead, pacemaker activity can be created by the overexpressed HCN4 gene in mature cardiomyocytes [24]. Studies have yet to report on the effect of the HCN2 or HCN4 gene on the differentiation of MSCs into cardiomyocytes. Therefore, this study has acquired MSCs successfully via in vitro porcine MSC isolation followed by flow cytometry for screening and identification. Therefore, HCN2 and HCN4 in MSCs were overexpressed and it was found that HCN2 and HCN4 could meaningfully improve in vitro MSC differentiation ability and restore the ionic current thereby, possibly indicating directional differentiation ability of MSCs in vitro could be improved under HCN2 and HCN4 combined action.

## 5. Conclusion

In summary, this experiment discovered that overexpressed HCN2 and HCN4 have the ability to moderately enhance in vitro differentiation of MSCs into cardiomyocytes therefore restoring MSC ionic currents. Results gained also suggest that overexpression of HCN2 and HCN4 genes can be present in the clinic and MSCs and differentiate directionally and transplanted into cardiomyocytes. However, immunosuppressive properties of MSCs, as well as higher viral infection risks, still need to be addressed in further studies.

## Figures and Tables

**Figure 1:** Porcine BMSC cell identification using flow cytometry. Isolated BMSCs were incubated with fluorescently labelled antibodies against CD90, CD44, CD45, and CD11B with flow cytometry used for detection.

**Figure 2:** BMSCs coexpressed HCN2 and HCN4. Immunofluorescence was used to detect expressed HCN2 and HCN4 in the cells. Green fluorescence indicates a positive expression of HCN2 while red fluorescence indicates a positive expression of HCN4. Magnification, 400x.

**Figure 3:** Induction of myocardial differentiation into BMSCs in vitro by HCN2 and HCN4. (a) Immunofluorescence staining was used to detect cardiomyocyte marker proteins *α*-actin and cTnT expression in cells; green fluorescence indicated the positive expression of *α*-actin while red fluorescence indicated the positive expression of cTnT. Magnification, 400x. (b) Western blot was used to detect the protein expression of *α*-actin, cTnT, and Desmin in cells. ^∗∗^*P* < 0.01 and ^∗∗∗^*P* < 0.001 vs. the BMSC group.

**Figure 4:** In vitro cultured BMSC ionic current could be restored by HCN2 and HCN4. (a) The HCN2+HCN4 group ionic current. (b) Ionic current post-CsCl treatment.

## Data Availability

All data generated or analyzed during this study are included in this article.
